The article "Decreased microRNA-182-5p helps alendronate promote osteoblast proliferation and differentiation in osteoporosis via the Rap1/MAPK pathway" was retracted in 2024. Reasons: plagiarized images; overlap with other authors' work; concerns about the data.

# Decreased microRNA-182-5p helps alendronate promote osteoblast proliferation and differentiation in osteoporosis via the Rap1/MAPK pathway

**DOI:** 10.1042/BSR20180696

**Published:** 2018-12-21

**Authors:** Bao-Long Pan, Zong-Wu Tong, Shu-De Li, Ling Wu, Jun-Long Liao, Yu-Xi Yang, Hu-Huan Li, Yan-Juan Dai, Jun-E Li, Li Pan

**Affiliations:** 1 Department of Laboratory, People’s Hospital of Yuxi City, Yuxi 653100, P.R. China; 2 Department of Nephrology, People’s Hospital of Yuxi City, Yuxi 653100, P.R. China; 3 Department of Biochemistry and Molecular Biology, School of Basic Medical Science, Kunming Medical University, Kunming 650500, P.R. China; 4 Department of Quality Management, Central Blood Station of Yuxi City, Yuxi 653100, P.R. China; 5 Department of Rehabilitation Medicine, People’s Hospital of Yuxi City, Yuxi 653100, P.R. China

**Keywords:** ADCY6, Alendronate, MicroRNA-182, Osteoporosis, Osteoblasts, Rap1/MAPK signaling pathway

## Abstract

Osteoporosis (OP) is a serious health problem that contributes to osteoporotic structural damage and bone fragility. MicroRNAs (miRNAs) can exert important functions over bone endocrinology. Therefore, it is of substantial significance to clarify the expression and function of miRNAs in bone endocrine physiology and pathology to improve the potential therapeutic value for metabolism-related bone diseases. We explored the effect of microRNA-182-5p (miR-182-5p) on osteoblast proliferation and differentiation in OP rats after alendronate (ALN) treatment by targeting adenylyl cyclase isoform 6 (ADCY6) through the Rap1/mitogen-activated protein kinase (MAPK) signaling pathway. Rat models of OP were established to observe the effect of ALN on OP, and the expression of miR-182-5p, ADCY6 and the Rap1/MAPK signaling pathway-related genes was determined. To determine the roles of miR-182-5p and ADCY6 in OP after ALN treatment, the relationship between miR-182 and ADCY6 was initially verified. Osteoblasts were subsequently extracted and transfected with a miR-182-5p inhibitor, miR-182-5p mimic, si-ADCY6 and the MAPK signaling pathway inhibitor U0126. Cell proliferation, apoptosis and differentiation were also determined. ALN treatment was able to ease the symptoms of OP. miR-182-5p negatively targeted ADCY6 to inhibit the Rap1/MAPK signaling pathway. Cells transfected with miR-182 inhibitor decreased the expression of ALP, BGP and COL I, which indicated that the down-regulation of miR-182-5p promoted cell differentiation and cell proliferation and inhibited cell apoptosis. In conclusion, the present study shows that down-regulated miR-182-5p promotes the proliferation and differentiation of osteoblasts in OP rats through Rap1/MAPK signaling pathway activation by up-regulating ADCY6, which may represent a novel target for OP treatment.

## Introduction

As a chronic systemic bone disease, osteoporosis (OP) manifests as less bone mass and a disorder of bone structure, which eventually contributes to the risk of fracture [1,2]. Changes in osteoblast or osteoclast production or the life span contribute to an imbalance between bone formation and resorption, which eventually results in OP [3]. According to statistics, fractures caused by OP will occur in individuals over 50 years old, among whom 50% are female and 20% are male; moreover, hip fracture is the most devastating because of the high rates of disability and mortality and the expensive costs, both to individuals and society as a whole [4]. By inhibiting phosphatase, alendronate (ALN) treatment is an effective anti-bone absorbent, which can promote the apoptosis of osteoclasts under the condition of extremely high doses [5]. China has approved a special formulation of ALN 70 mg/vitamin D3 5600 IU (ALN/D5600) considering that patients with OP can cure their disease and absorb sufficient vitamin D at the same time [6]. Although ALN is highly recommended in international treatment, the accompanying side effects cannot be ignored, for example, weight loss, sciatica, rash and asthma [7]. Moreover, in the differentiation of bone cells, microRNAs (miRNAs) serve irreplaceable functions, regulating the lineage commitment and cell progression of mesenchymal stem cells [8].

As a member of the miR-183–182 cluster that encodes miR-96, miR-182 and miR-183, MiR-182 plays an important role in regulating the apoptosis, growth and differentiation of cells [9,10]. Adenylyl cyclase isoform 6 (ADCY6) is one of the colon membrane-bound isoforms of adenylyl cyclase, and it has been shown to participate in elevated blood pressure and the cardiovascular response [11]. Rap1, a small GTP-ase, dynamically controls the coordination of cell spreading and endothelial barrier function by regulating cell–cell adhesion, cell–matrix adhesion and actin rearrangement [12]. Based on the activation of Rap1, the excitability of neuronal and cocaine-induced behavioral reward responses can be induced through the mitogen-activated protein kinase (MAPK)/extracellular signal-regulated kinase (ERK) pathway [13]. The MAPK/ERK signaling code also functions as a more common original cancer signal with the exception of a tumor suppressor according to recent evidence [14]. However, research regarding the connection between miR-182-5p and the Rap1/MAPK signal pathway and its controlling function in OP remains limited. In the present study, we will explore the mechanism of the miR-182-5p, ADCY6 and Rap1/MAPK signaling pathway in osteoblast proliferation and differentiation in OP rats after ALN treatment. We aim to provide a new basis for the development of targeted therapy for OP.

## Methods

### Ethics statements

The present study was carried out in strict accordance with the recommendations in the Guide for the Care and Use of Laboratory Animals of the National Institutes of Health. The protocol was approved by the Institutional Animal Care and Use Committee of People’s Hospital of Yuxi City.

### Model establishment and specimen collection

Rats were fed adaptively for 1 week during which there was no death. Thirty rats were randomly divided into sham (with no treatment) group, operation group (OP group) and ovariectomy + ALN sodium treatment (ALN group) with 10 rats per group (ALN sodium was purchased from Yangtze River Pharmaceutical Group, Taizhou, Jiangsu, China). The OP model was established in the OP group and the ALN group via bilateral ovariectomies [15]. Fasting for 12 h before surgery, 3% pentobarbital sodium (1 ml/kg) was injected into the abdominal cavity of the rats for anesthesia. The abdominal region was fixed to a surgical board, and a dorsal approach was used under sterile conditions. A longitudinal incision was subsequently made (1 cm) in the central back to separate the skin from both sides. The dorsal muscles were incised on either side of the spine (incision should be as small as possible) with the aim to separate the cellulite. The stump was ligated by a surgical line after the exposed pink ovaries were removed. After releasing the hemostatic forceps and gently placing the uterus into the abdominal cavity, the muscle layer and skin were sutured, respectively. The incision was subsequently cleaned using an alcohol cotton ball, the other ovary was removed and the wound was sutured as previously described. The ovaries of the rats in the sham group were only exposed and were not removed. Only a small amount of surrounding adipose tissues was removed and sutured. A gentamycin sulfate injection was continuously administered into the muscle to resist infection 3 d after the operation. One week after the model was successfully established, the ALN sodium was crushed at a dosage of 0.1 mg kg^−1^ d^−1^ [16] and prepared in a suspension with distilled water. The rats in the ALN group were subsequently fed the suspension. The rats in the sham group and the OP group were administered normal saline for 4 weeks continuously.

After 4 weeks of drug treatment, the rats in each group were fasted for 12 h with water deprivation for 6 h. The abdominal cavities were injected with 3% pentobarbital sodium (1 ml/kg). Blood was collected from the femoral artery and centrifuged at 2863 × *g* for 10 min to separate the serum. The femurs were separated, and the left femurs were rapidly removed. After being washed with normal saline, the left femurs were stored in liquid nitrogen, and the right femurs were fixed with 10% formalin.

### Determination of blood phosphorus, serum calcium and bone mineral density

The fresh left femur after isolation was arranged on the test board and scanned by a dual energy X-ray bone densitometer (HOLIGIC QDR-4500w, Waltham, MA, USA). Software was employed to analyze the bone mineral density (BMD) of the whole femur using the small animal model during the scanning. Rat serum was extracted, and the calcium and phosphorus levels were determined by an automatic biochemical analyzer (TBA-30, Toshiba, Otawara, Japan), in which the serum calcium was tested by the alkaline picrate method, and the blood phosphorus were verified via direct ultraviolet spectrophotometry.

### Hematoxylin–eosin (HE) staining and immunohistochemistry

Femur tissues fixed with 10% formaldehyde were decalcified in 10% nitric acid solution and then washed overnight, embedded in paraffin wax and cut into 4 μm sections. The sections were subsequently placed in the oven at 65 °C for 6 h. The sections were conventional dewaxed, washed for 1–2 min, stained with hematoxylin for 3–6 min and then washed under running water for 1–2 min. The sections were combined with 1% hydrochloric acid ethanol for 1–3 s, slightly washed for 1–2 s, returned to blue with ammonia for 5–10 s, washed for 15–30 s and stained by 0.5% eosin solution for 2–3 min. The sections were washed with distilled water again for 1–2 s, dehydrated sequentially in 80%, 95% and 100% ethanol for 15–30 s, 15–30 s and 1–2 s, respectively, cleared with xylenes (xylene I/II) for 2–3 s each and then sealed by neutral gum. The HE staining of the femoral tissues in each group was observed under an optical microscope (B561T-PH2-J11, Olympus Optical Co., Ltd., Tokyo, Japan), and the microphotograph (×400) was performed. The HE staining results were quantified with ImageJ Software. The paraffin sections of the femur tissues of the rats were prepared (steps were performed as previously described), blocked with 5–10% normal goat serum [diluted with phosphate buffered saline (PBS)] and incubated at room temperature for 10 min. The serum was discarded without washing. The sections were combined with a proper proportion of diluted primary, rabbit antibody to CD34 antibody (1:200, ab81289) and rabbit antibody to receptor activator of nuclear factor-kappa B (RANK, 1:200, ab216484) and incubated at 37°C for 12 h or 4°C overnight. The antibodies were purchased from Abcam Inc. (Cambridge, MA, USA). Following three washes in PBS for 5 min each, the sections were stained with diaminobenzidine (DAB). The sections were then fully washed with tap water, counterstained and sealed.

### TdT-mediated dUTP-biotin nick end-labeling assay

The apoptosis of osteoblasts was observed by staining with the TdT-mediated dUTP-biotin nick end-labeling (TUNEL) kit (C1086, Beyotime Biotechnology Co., Ltd., Shanghai, China). Ten percent formaldehyde fixed femoral tissues were embedded in paraffin, cut into sections and dewaxed with conventional paraffin. The sections were subsequently rehydrated with gradient alcohol and soaked in 3% H_2_O_2_ solution at room temperature for 10 min. After being washed with PBS for 5 min, the sections were combined with 50 μl of 20 μg/ml proteinase K (P6556, Sigma–Aldrich Chemical Company, St Louis, MO, USA) solution and hydrolyzed at room temperature for 20 min to remove tissue protein. The sections were washed three times with PBS (5 min each time) and combined with citrate buffer for antigen retrieval for 30 min. The sections were subsequently washed two times with PBS (5 min each time). TdT enzyme reaction solution (50 μl) was added to the sections and placed in a wet box at 37°C for 1 h under conditions void of light. The TdT enzyme-free reaction solution was used as the negative staining control. After three washes with PBS (5 min each time), the sections were combined with 50 μl of peroxidase-labeled anti-digoxigenin and placed in a wet box at 37°C for 30 min under conditions void of light. After three washes with PBS (5 min each time), the sections were combined with 4′,6-diamidino-2-phenylindole (DAPI) solution (C1002, Beyotime Biotechnology Co., Shanghai, China) to develop at room temperature for 10 min. After two washes with PBS (5 min each time), the sections were mounted with neutral gum, and a fluorescence microscope (BX53, Olympus Optical Co., Ltd., Tokyo, Japan) was used for observation and photograph. The nuclei of positive apoptotic cells were stained with green, and those of the normal cells were stained with blue. Ten views were randomly selected to count the ratio of the positive cells to the total number of cells as the apoptosis index (AI).

### Reverse transcription quantitative polymerase chain reaction (RT-qPCR)

The left femurs were grinded into homogenate. Total RNA from the femur tissues was extracted according to the instructions of the Trizol kit (15596-026, Invitrogen, Gaithersburg, MD, USA). A nucleic acid and protein analyzer (BioPhotometer D30, Eppendorf, Hamburg, Germany) was used to measure the RNA purity. RNA was reversely transcripted into cDNA using the reverse transcription kit (K1621, Fermentas, Maryland, N.Y., USA). The primer sequences of miR-182-5p, ADCY6, extracellular signal-regulated kinase 1/2 (ERK1/2), P38 MAPK, proliferating cell nuclear antigen (PCNA), Ras-related protein 1 (Rap1), bone morphogenetic protein-2 (BMP2), bone gla protein (BGP), alkaline phosphatase (ALP), type I collagen (COL IA1), U6 and β-actin (Table 1) were synthesized by Shanghai Genechem Co., Ltd. (Shanghai, China). A fluorescent quantitative PCR Kit (Takara, Dalian, Liaoning, China) was used to determine the mRNA levels of the genes, and the reaction system was: 5.3 µl of 2 × Taq Master Mix, 1 µl of forward primer (5 µM), 1 µl of reverse primer (5 µM), 1 µl of cDNA and 11.7 µl of RNase Free H_2_O. The reaction conditions were as follows: predenaturation at 95°C for 5 min, a total of 40 cycles for the denaturation at 94°C for 45 s, anneal at 56°C for 45 s and extension at 72°C for 45 s. A real-time fluorescence quantitative PCR instrument (ABI 7500, ABI, Foster City, CA, USA) was applied for measurement. U6 served as the internal control of miR-182-5p, and β-actin was the internal control of the other related genes. The relative expression of each target gene was calculated based on the 2^−ΔΔCt^ method, and each experiment was repeated three times. The expression of mRNA: ΔΔCt [Ct _(target gene of the experimental group)_ − Ct _(internal control of the experimental group)_] − [Ct _(target gene of the NC group)_ − Ct _(internal control of the NC group)_], the relative transcription level of mRNA = 2^−ΔCt^.

**Table 1:** The primer sequences for RT-qPCR

Gene	Sequence
miR-182-5p	F: 5′-GGGTCTAGCTGCCGGAGG-3′
	R: 5′-CGGTGTGAGTTCTACCATTGC-3′
U6	F: 5′-GCTCGCTTCGGCAGCACA-3′
	R: 5′-GAGGTATTCGCACCAGAGGA-3′
ADCY6	F: 5′-CAGCAGGGTAGTGTGTGCAG-3′
	R: 5′-TCTGCATTTGATTTTGGCCT-3′
ERK1/2	F: 5′-CTCAAGCCTTCCAACCTC-3′
	R: 5′-TTCCACGGCACCTTATTT-3′
P38 MAPK	F: 5′-GCATAAAGCCCAAGAGAACCAAC-3′
	R: 5′-GACAGGACAAGCTCCAGAGCACA-3′
Rap1	F: 5′-GCGTCTGGTCA GAGAGCTG-3′
	R: 5′- TCAATCCTCCGAGCTACATTCT-3′
β-actin	F: 5′-GGCACCACACTT TCTACAAT-3′
	R: 5′-AGGTCTCAAACATGATCTGG-3′
PCNA	F: 5′-CGGCGTGAACCTACAGA-3′
	R: 5′-TCGCAGCGGTATGTGTCGAA-3′
BMP2	F: 5′-ACGATGCCGCCATTTGTG-3′
	R: 5′-CGCCTCGCCTTCTTCAGT-3′
BGP	F: 5′-AGCGACTCTGAGTCTGACAAA-3′
	R: 5′-AACGGTGGTGCCATAGATGCG-3′
ALP	F: 5′-CAGTGGTATTGTAGGTGCTGTG-3′
	R: 5′-TTTCTGCTTGAGGTTGAGGTTAC-3′
COL1A1	F: 5′-GTCCTATGGCTATGATGAGAAATC-3′
	R: 5′-CACCATCCAAACCACTGAAAC-3′

Abbreviations: ADCY6, adenylate cyclase 6; ALP, alkaline phosphatase; BGP, bone gla protein; BMP2, bone morphogenetic protein-2; COL I, type I collagen; ERK1/2, extracellular signal-regulated kinase 1/2; F, forward; miR-182-5p, microRNA-182-5p; PCNA, proliferating cell nuclear antigen; R, reverse; Rap1, Ras-related protein 1; RT-qPCR, quantitative real-time polymerase chain reaction.

### Western blot analysis

Left femur tissue samples (50 mg) were cut into pieces, combined with protein lysate (R0010, Beijing Solabio Life Sciences Co., Ltd., Beijing, China), lysed and centrifuged, and the supernatant was collected to determine the protein concentration. Total protein was separated via 10% sodium dodecyl sulfate polyacrylamide gel electrophoresis (P1200, Beijing Solabio Life Sciences Co., Ltd., Beijing, China), transferred to a polyvinylidene fluoride (PVDF) membrane (HVLP04700, Millipore, Bedford, MA, USA) using the semidry transfer method, and stained with Ponceau S (P0012, Beijing Solabio Life Sciences Co., Ltd., Beijing, China) to observe protein transfer. The membrane was subsequently washed two times with Tris-buffered saline with Tween 20 (TBST), blocked at room temperature for 2 h in 5% skimmed milk powder and washed three times with TBST. The membrane was then incubated with the following primary antibodies overnight at 4°C: anti-rabbit ADCY6 (1:500, ab14718), anti-rabbit ERK1/2 (1:1000, ab17942), anti-rabbit P38 MAPK (1:1000, ab197348), anti-rabbit Rap1 (1:1000, ab92836), anti-rabbit PCNA (1 µg/ml, ab18197), anti-rabbit BMP2 (1:500, ab14933), anti-rabbit BGP (1:1000, ab93876), anti-rabbit ALP (1:500, ab83259), anti-rabbit COL I (1:1000, ab34710) and anti-rabbit β-actin (1:1000, ab8227) (Abcam, Cambridge, MA, UK), as well as the anti-rabbit p-ERK and anti-rabbit p-P38 MAPK (1:2000, 4370; 1:1000, 4511, Cell Signaling Technology, Beverly, MA, USA). After being rinsed with TBST three times (10 min per time), the membrane was incubated with horseradish peroxidase (HRP)-labeled secondary goat anti-rabbit IgG (1:2000, ab6721, Abcam, Cambridge, MA, UK) at room temperature for 2 h and then washed three times (10 min each time) with TBST. DAB reaction solution was used to develop the color. A gel imager (Gel Doc XR, Bio-Rad, Hercules, CA, USA) was used for photograph, and the ratios of the gray values of the target bands to the internal reference bands serve as the relative protein expression levels. This method was also suitable for the determination of the protein levels in the cell experiment.

### Osteoblast isolation, culture and identification

Left femur tissues of the OP group were obtained. The blood vessels and connective tissues were cleaned, placed in 1 ml of PBS, cut into 1 mm³ tissue blocks, washed two times with PBS and centrifuged. With the PBS aspirated, cells were combined with 5 ml of 0.25% trypsin solution for 20 min in a 37°C water bath, followed by the addition of 5 ml of 0.1% collagen II. Cells were then detached in a 37°C water bath for 60 min. M199 culture medium (3 ml, 31100035, Gibco, Carlsbad, CA, USA) that contained 10% fetal bovine serum (FBS, 16000-044, Gibco, Carlsbad, CA, USA) was added to the cells. Following centrifugation for 10 min at 179 × *g*, the supernatant was removed. The cells were subsequently combined with 3 ml of M199 culture medium that contained 10% FBS for cell resuspension and incubated in a 5% CO_2_ incubator (ZXKR-1150, Shanghai Zhicheng Analytical Instrument Manufacturing Co., Ltd., Shanghai, China) at 37°C. After 24 h, the medium was changed for the first time; the medium was subsequently changed every 2–3 d. The third generation of cells in the logarithmic growth phase was used in this experiment, and the cell morphology was observed under an inverted microscope (IX53, Olympus Optical Co., Ltd., Tokyo, Japan).

#### ALP staining

After the third generation of cell detachment and culture, 5-bromo-4-chloro-indolyl-phosphatase (BCIP) and the ALP assay kit (Nanjing Jiancheng Biology Company, Nanjing, Jiangsu, China) were used for staining. After being fixed with formalin, the cell samples were washed three times with PBS solution (3 min each time). The proper amounts of BCIP and BI staining solution (which contained 3 ml of ALP staining buffer, 10 ml of BCIP solution and 20 ml of nitroblue tetrazolium) were added to fully cover the sample. After incubating in conditions void of light at room temperature for 2 h, BCIP was removed and BI staining solution was added. Next, 1–2 times distilled water washes were conducted to terminate the color development, and the sample was observed under a fluorescence microscope (BX53, Olympus Optical Co., Ltd., Tokyo, Japan).

#### Calcium nodules staining (alizarin red staining)

The third generation of cells were cultured for two weeks and then mineralized to form opaque calcified nodules. The cell samples were washed 1–2 times with PBS, fixed with 95% ethanol for 10 min, washed 1–2 times with PBS again, covered and stained with 0.1% alizarin red solution for 10 min, rinsed with PBS and observed under an inverted microscope.

### Cell transfection and grouping

The third generation of femoral osteoblasts extracted from the OP group were allocated into eight groups: blank (no transfected plasmid), negative control (NC, transfected with NC plasmid), miR-182-5p mimic (transfected with miR-182-5p mimic plasmid), miR-182-5p inhibitor (transfected with miR-182-5p inhibitor plasmid), U0126 group (treated with U0126), miR-182-5p inhibitor + U0126 group (transfected with miR-182-5p inhibitor plasmid and treated with U0126), siRNA-ADCY6 (transfected with ADCY6 interference plasmid) and miR-182-5p inhibitor + si-ADCY6 (cotransfected with miR-182-5p and ADCY6 interference plasmid). After being detached with 0.25% trypsin, cells were resuspended with M199 culture medium that contained 10% FBS to adjust the density to 1 × 10^5^ cells/ml and seeded in a 6-well plate. When the confluence of the cells reached 70%, the culture medium was replaced with serum-free M199 culture medium, and cells were transfected after 24 h of culture. Lipofectamine 2000 (6 µl, 11668-019, Invitrogen Inc., Carlsbad, CA, USA) was diluted in 200 μl of serum-free Opti-MEM medium (31985070, Gibco, Carlsbad, CA, USA), and 2 μg of target plasmid were diluted in 100 μl of serum-free Opti-MEM medium, mixed respectively and cultured at room temperature for 10 min. These two solutions were mixed together and incubated for 20 min at room temperature. The culture medium in the six-well plate was aspirated, and 1.7 ml of serum-free M199 culture medium was added to each well; the transfected compound was added to the corresponding wells. The final concentration of U0126 treated cells was 10 µM [17]. After being incubated for 18 h in a 5% CO_2_ incubator at 37°C, fresh complete medium was replaced, and cells were collected after transfection for 48 h.

### Dual-luciferase reporter gene assay

According to the online prediction website microRNA.org, the target gene of miR-182-5p was predicted. Whether ADCY6 was a direct target of miR-182-5p was identified via a dual-luciferase reporter gene assay. Endonuclease sites (SpeI and HindIII) were introduced into the pMIR-reporter to design complementary mutation sites of seed sequences on the wild type (WT) ADCY6. The target fragment was inserted into the pMIR-reporter plasmid using T4 DNA ligase after restriction endonuclease digestion. Correctly sequenced luciferase-reporter plasmid WT or mutated (MUT) were cotransfected into HEK-293T cells (CRL-1415, Shanghai Xin Yu Biotech Co., Ltd, Shanghai, China) with miR-182-5p, respectively. After transfection for 48 h, the culture medium was discarded and washed two times with PBS; the cells were then collected and lysed. The activity of luciferase was tested using the luciferase reporter gene detection system (Dual-Luciferase^®^ Reporter Assay System, E1910, Promega Corporation, Madison, WI, USA). The activity of firefly luciferase was measured by the addition of 50 μl of firefly luciferase solution into every 10 μl of sample. Then, 50 μl of Renilla luciferase solution were added to evaluate the activity of Renilla luciferase; the ratio of the firefly luciferase activity to the Renilla luciferase activity was the relative luciferase activity. The experiment was repeated three times.

### 3-(4,5-Dimethylthiazol-2-yl)-2,5-diphenyltetrazolium bromide assay

Each transfected group of osteoblasts in the logarithmic growth period was inoculated into 96-well plates at a density of 1 × 10^4^ cells/well, with eight replicates in each group. There was a blank well that contained only medium without cells. When the cell confluence reached 70%, 10 μl of 5 mg/ml 3-(4,5-dimethylthiazol-2-yl)-2,5-diphenyltetrazolium bromide (MTT) reagent (ST316, Shanghai Beyotime Biotechnology Co., Ltd., Shanghai, China) were added to each well, and the cells were cultured in a 5% CO_2_ incubator at 37°C for 4 h. With the supernatant aspirated, the 96-well plate was washed one time with PBS, and 100 µl of dimethyl sulfoxide (DMSO, D5879, Sigma–Aldrich Chemical Company, St Louis, MO, USA) were added to each well. The 96-well plate was subsequently vibrated at a low speed on the shaking table for 10 min. The optical density (OD) at 490 nm was measured using a microplate reader (MK3, Thermo, Pittsburgh, PA, USA) for each well. Cell survival rate = (OD value of the experiment well − OD value of the blank well)/OD value of blank well. The experiment was conducted three times to obtain the mean value.

### Detection of ALP and osteocalcin secretion

The *P*-nitrophenyl phosphate (PNPP) method was used to determine the ALP content: third generation osteoblasts in the ALN group were seeded in a 12-well plate with a density of 1 × 10^5^ cells/ml and combined with 250 μl of 0.05% TritnoX-100 for cell lysis. Cell lysates (50 μl) were transferred to a 96-well plate, combined with 50 μl of 4.5 mmol/l PNPP (Am- resco, Solon, OH, USA) and water-bathed at 37°C for approximately 30 min. Finally, 50 μl of 0.1 mol/l sodium hydroxide were added to terminate the reaction. The absorbance (*A*) value at 405 nm was measured using a microplate reader (Bio-Rad, Inc., Hercules, CA, USA). Cell lysates (20 μl) were extracted in each well and combined with 180 μl of Coomassie staining solution (Sigma–Aldrich Chemical Company, St Louis, MO, USA). The value at 595 nm was measured using a microplate reader. Total protein (mg/l) was obtained according to the standard curve of protein.

Osteocalcin secretion measurement: third generation osteoblasts from the ALN group were seeded in a 48-well plate with a density of 2 × 10^4^ cells/ml (0.5 ml each well). After 24 h, the cells were cultured in Dulbecco’s Modified Eagle’s Medium (DMEM, Gibco, Carlsbad, CA, USA) that contained 10% calf serum (0.45 ml each well) and incubated in a 5% CO_2_ incubator (ZXKR-1150, Shanghai Zhicheng Analytical Instrument Manufacturing Co., Ltd., Shanghai, China) at 37°C. When the cell confluence reached 80%, the serum-containing medium was replaced with serum-free bovine serum albumin (BSA) culture medium (Gibco, Carlsbad, CA, USA). After 3 d of culture, the cell culture medium was collected. The osteocalcin secretion was obtained according to the instructions of the osteocalcin radioimmunoassay kit (Beijing East Asia Immunological Technology Institute, Beijing, China).

### Flow cytometry

With transfection for 48 h, the culture medium was discarded, and the cells were washed one time with PBS. The cells were treated with 0.25% trypsin. Cells were collected and centrifuged at 179 × ***g*** for 5 min at 4°C. The supernatant was removed, and the cells were washed two times using PBS and centrifuged at 179 × ***g*** for 5 min. The supernatant was discarded, and the cells were fixed with precooled 70% ethanol at 4°C overnight. The cells were rinsed with PBS, centrifuged again at 179 × ***g*** for 5 min and incubated with 10 µl of RNase enzyme at 37°C for 5 min. Following the addition of 1% propidium iodide (PI) staining buffer (40710ES03, Shanghai QCbio Science & Technologies Co., Ltd., Shanghai, China) under conditions void of light for 30 min, the samples were analyzed using a flow cytometer (Becton, Dickinson and Company, Franklin Lakes, NJ, USA) to detect the cell cycle by red fluorescence at an excitation wavelength of 488 nm. The experiment was repeated three times.

After transfection for 48 h, cells were detached with ethylenediaminetetraacetic acid (EDTA)-free trypsin and collected in a flow tube, followed by centrifugation at 4°C, 179 × ***g*** for 5 min. The supernatant was discarded, and the cells were washed with precooled PBS and centrifuged again at the speed of 179 × ***g*** for 5 min. An Annexin-V-fluorescein isothiocyanate (FITC)/PI apoptosis detection kit (CA1020, Beijing Solabio Life Sciences Co., Ltd, Beijing, China) was used to detect the apoptosis of cells after the supernatant was discarded. Binding buffer was used to wash cells. The cells were resuspended in a mixed solution (Annexin-V-FITC and binding buffer at a ratio of 1:40), incubated at room temperature for 30 min, and combined with mixed solution (PI and Binding buffer at a ratio of 1:40). The cells were incubated at room temperature for 15 min. The flow cytometer was used to detect the cell apoptosis. The lower left quadrant showed living cells as Annexin V−/PI−, and the right upper quadrant was the advanced apoptotic cell or the secondary necrosis cell as Annexin V+/PI+, while the right lower quadrant was the early apoptotic cell as Annexin V+/PI−. The experiment was repeated three times.

### Statistical analysis

Statistical analyses were conducted using SPSS 21.0 statistical software (IBM Corp., Armonk, N.Y., USA). Measurement data are expressed as the mean ± standard deviation. Multiple groups were compared by one-way analysis of variance. *P* < 0.05 indicated that the difference was statistically significant.

## Results

### ALN significantly enhances BMD and serum calcium while decreasing serum phosphorus in OP

After 4 weeks of the drug intervention, there was no death of rats. The content of the serum calcium, blood phosphorus and BMD were determined. There were significant differences in the blood phosphorus and BMD between the OP group and the sham group. Compared with the OP group, the ALN group had a significantly increased BMD, showing its therapeutic effect. Compared with the sham group, the OP and ALN groups had increased serum calcium (*P* > 0.05) and significantly decreased blood phosphorus content and BMD (*P* < 0.05). Compared with the OP group, the ALN group had increased serum calcium and decreased serum phosphorus with no significant difference (*P* > 0.05), as well as a significantly increased BMD (*P* < 0.05). ALN treatment could elevate the BMD (Table 2).

**Table 2:** ALN significantly increased serum calcium, decreased serum phosphorus and enhanced BMD in OP

Group	Serum calcium (mmol/l)	Serum phosphate (mmol/l)	Bone mineral density (g/cm^3^)
Sham	2.47 ± 0.15	2.75 ± 0.26	1.53 ± 0.07
OP	2.54 ± 0.18	2.36 ± 0.25*	1.03 ± 0.06*
ALN	2.52 ± 0.20	2.44 ± 0.31*	1.31 ± 0.05^*#^

Abbreviations: ALN, alendronate; OP, osteoporosis. *, *P* < 0.05 *vs.* the sham group; #, *P* < 0.05 *vs.* the OP group.

### ALN treatment alleviates the pathological changes of femoral tissue in OP

HE staining was used to observe the pathological changes of femoral tissue in OP. The trabecular trabeculae were thick and well-arranged into mesh, with a small gap, deep coloring, complete shape and structure, density of bone trabeculae, normal area and a relatively small medullary cavity in the sham group. In the OP group, the trabecular bone was thinner, cortical thinning was observed, and the morphological structure was poor with a break. The gap between the trabecular increased, the bone density and area were reduced, the number of hematopoietic cells decreased, the fat vacuole was elevated, the osteoblasts decreased and the osteoclasts increased, which are typical osteoporotic signs, indicating that the model was successfully established. In the ALN group, there was no obvious thinning of the cortical bone and no obvious thinning of the trabecular bone with normal trabecular connectivity. The gap between the trabecular enlarged slightly, the area of the trabecular space did not significantly decrease, the number of hematopoietic cells in the medullary cavity was elevated and the osteoclasts decreased (Figure 1A). The expression of CD34 and RANK was determined by immunohistochemistry, and positive expression was identified as yellow or brown granules on the cell membrane (Figure 1B). The statistical results showed that the positive expression of the hematopoietic marker CD34 in the OP group was lower than that in the sham group, while the positive expression of the osteoclast marker RANK was increased. Compared with the OP group, the ALN group showed increased expression of the hematopoietic marker CD34 and decreased expression of the osteoclast marker RANK (Figure 1C).

**Figure 1:** ALN treatment significantly improves OP symptoms (**A**) HE staining (40×) shows the effect of ALN treatment on the histopathological changes of femoral tissues in rats; (**B**) immunohistochemical staining of CD34 and RANK in the sham, OP and ALN groups (400×); ALN, alendronate; HE, hematoxylin–eosin; OP, osteoporosis; RANK, receptor activator of NF-KappaB.

### ALN treatment inhibits the apoptosis of cells in femoral tissue in OP

TUNEL staining was applied for cell apoptosis determination. The positive cells of apoptosis were stained with dark brown. The AI of the femur tissues in the sham group was (24.35 ± 2.89)%. The AI of the femur tissues in the ALN group was significantly lower (25.8 ± 2.97)% than that of the OP group (44.9 ± 4.53)% (*P* < 0.05). ALN treatment could inhibit the apoptosis of cells in rats with OP (Figure 2).

**Figure 2:** ALN treatment decreases cell apoptosis in OP (**A**) TUNEL staining reflects apoptotic cells (400 ×); (**B**) AI of femoral tissues; *, *P* < 0.05 *vs.* the sham group, #, *P* < 0.05 *vs.* the OP group; ALN, alendronate; OP, osteoporosis; TUNEL, TdT-mediated dUTP-biotin nick end-labeling assay; AI, apoptosis index.

### MiR-182-5p is down-regulated, whereas ADCY6 is up-regulated and the Rap1/MAPK signaling pathway is activated after treatment with ALN

The miR-182-5p expression and the mRNA and protein levels of ADCY6 and the Rap1/MAPK signaling pathway-related factors in femoral tissues were determined by RT-qPCR (Figure 3A) and Western blot analysis (Figure 3B,C). Compared with the sham group, the OP group had a significantly higher expression of miR-182-5p, whereas it had significantly down-regulated mRNA and protein levels of ADCY6, ERK1, ERK2, Rap1 and P38 MAPK, as well as the extent of ERK1/2 and P38 MAPK phosphorylation (all *P* < 0.05). Compared with the OP group, the ALN group had a decreased expression of miR-182-5p and increased mRNA and protein levels of ADCY6, ERK1, ERK2, Rap1 and P38 MAPK, as well as the extent of ERK1/2 and P38 MAPK phosphorylation. It was determined that miR-182-5p was highly expressed in the rats with OP, while ADCY6, ERK1, ERK2 and Rap1, as well as the extent of ERK1/2 and P38 MAPK phosphorylation were lowly expressed. The ALN group showed the opposite trend, indicating that it has an inhibitory effect on rats with OP.

**Figure 3:** MiR-182-5p is up-regulated, whereas ADCY6 and the Rap1/MAPK signaling pathway are inhibited after treatment with ALN (**A**) miR-182-5p expression and mRNA levels of ADCY6, ERK1, ERK2, Rap1 and P38 MAPK in response to ALN treatment; (**B**) the gray value of ADCY6, ERK1/2, p-ERK1/2, P38 MAPK, p-P38 MAPK and Rap1 protein bands in response to ALN treatment; (**C**) protein levels of ADCY6, ERK1/2, Rap1 and P38 MAPK and the extent of ERK1/2 and P38 MAPK phosphorylation in response to ALN treatment; *, *P* < 0.05 *vs*. the sham group; #, *P* < 0.05 *vs*. the OP group. MiR-182-5p, microRNA-182-5p; OP, osteoporosis; ADCY6, adenylate cyclase 6.

### Osteoblasts are successfully cultured

Microscopic observation showed that the osteoblasts were triangular or multispindle and the cells were morphologically diverse after several days. The osteoblasts were spindle shaped, triangular or polygonal, with protuberance. The nuclei were round or oval. In the growth stage, cell division was more common, and the cells were multiple and connected. At the time of confluence, the cells are stony and could be overlapped. The overlapping cells gradually formed cell nodules, followed by collagenous accumulation and calcium salt deposition, and finally formed an opaque mineralized nodule (Figure 4A). Alkaline phosphatase staining showed that most cells were colored (black or gray). The cytoplasm showed a positive reaction of gray-black granule or block deposit (Figure 4B). Calcium nodule staining (alizarin red staining): typical orange calcified nodules were shaped (Figure 4C). These results were consistent with the characteristics of osteoblasts, which can be used to verify the success of the osteoblast culture.

**Figure 4:** Osteoblasts are cultured successfully (**A**) The morphology of osteoblasts (the original magnification is 100×); (**B**) ALP images of osteoblasts (the original magnification is 200×); (**C**) alizarin red staining images of osteoblasts (original magnification is 100×). ALP, alkaline phosphatase staining.

### ADCY6 is a direct target gene of miR-182-5p

According to the online prediction website analysis, there is a binding site between miR-182-5p and ADCY6 3′UTR, and ADCY6 is the target gene of miR-182-5p (Figure 5A). Dual-luciferase reporter gene assays were used to verify that ADCY6 is the target of miR-182-5p (Figure 5B). Compared with the NC group, the miR-182-5p mimic group significantly inhibited the activity of luciferase in the ADCY6-WT 3′UTR (*P* < 0.05), while miR-182-5p had no significant effect on the activity of luciferase in the MUT 3′UTR (*P* > 0.05). MiR-182-5p could specifically bind to ADCY6 3′-UTR, and ADCY6 is the target gene of miR-182-5p.

**Figure 5:** ADCY6 is the target gene of miR-182-5p (**A**) Binding regions between ADCY6 3′UTR and miR-182-5p sequence according to the online prediction website analysis; (**B**) luciferase activity of the ADCY6 Wt and ADCY6 Mut after transfection; *, *P* < 0.05 *vs*. the NC group. ADCY6, adenylate cyclase 6; NC, negative control; miR-182-5p, microRNA-182-5p.

### MiR-182-5p inhibits the expression of ADCY6 and the Rap1/MAPK signaling pathway activation

RT-qPCR (Figure 6A) and Western blot analysis (Figure 6B,C) were conducted to measure the expression of miR-182-5p, ADCY6 and the Rap1/MAPK signaling pathway-related genes after transfection. There was no significant difference in the gene expression in the NC group compared with the blank group (*P* > 0.05). Compared with the blank and NC groups, the miR-182-5p mimic group showed promoted miR-182-5p expression, and the miR-182-5p mimic and si-ADCY6 groups had down-regulated mRNA and protein levels of ADCY6, ERK1, ERK2, P38 MAPK and Rap1, as well as the extent of ERK1/2 and P38 MAPK phosphorylation (all *P* < 0.05). The expression of miR-182-5p in the miR-182-5p inhibitor group was down-regulated, and the mRNA and protein levels of ADCY6, ERK1, ERK2, P38 MAPK and Rap1, as well as the extent of ERK1/2 and P38 MAPK phosphorylation were up-regulated in the miR-182-5p inhibitor group (all *P* < 0.05). The expression of miR-182-5p was down-regulated in the miR-182-5p inhibitor + si-ADCY6 group with no other significant difference (*P* > 0.05). After the addition of the signal transduction pathway inhibitor U0126, the expression trend of the related signal transduction protein was similar to that of the miR-182-5p mimic group and the si-ADCY6 group. The ADCY6 expression was enhanced; however, there was no difference in the expression of the related signal transduction protein between the miR-182-5p inhibitor + U0126 group and the blank group. MiR-182-5p could reduce the expression of ADCY6, thus suppressing the activation of the Rap1/MAPK signaling pathway.

**Figure 6:** MiR-182-5p inhibits the expression of ADCY6 and suppressed the Rap1/MAPK signaling pathway (**A**) The expression of miR-182-5p and mRNA levels of ADCY6, ERK1, ERK2, P38 MAPK and Rap1 in response to the treatment of miR-182-5p mimic, miR-182-5p inhibitor, si-ADCY6, miR-182-5p inhibitor + si-ADCY6, U0126 or miR-182-5p inhibitor + U0126; (**B**) the gray value of ADCY6, ERK1/2, p-ERK1/2, P38 MAPK, p-P38 MAPK and Rap1 protein bands in response to the treatment of miR-182-5p mimic, miR-182-5p inhibitor, si-ADCY6, miR-182-5p inhibitor + si-ADCY6, U0126 or miR-182-5p inhibitor + U0126; (**C**) protein levels of ADCY6, ERK1,/2, Rap1 and P38 MAPK and the extent of ERK1/2 and P38 MAPK phosphorylation in response to the treatment of miR-182-5p mimic, miR-182-5p inhibitor, si-ADCY6, miR-182-5p inhibitor + si-ADCY6, U0126 or miR-182-5p inhibitor + U0126; *, *P* < 0.05 *vs*. the blank and NC groups; #, *P* < 0.05 *vs*. the miR-182-5p inhibitor group; OP, osteoporosis; ADCY6, adenylate cyclase 6; Rap1, Ras-related protein 1; MAPK, mitogen-activated protein kinase; ERK, extracellular signal-regulated kinase; miR-182-5p, microRNA-182-5p.

### Down-regulation of miR-182 promotes osteoblast proliferation

MTT assay and Western blot analysis were employed to evaluate the osteoblast proliferation (Figure 7A) and PCNA protein level, respectively (Figure 7B,C). The OD values of the cells in each group were all increased with time. There was no difference in the PCNA protein level and OD values between the blank and NC groups (*P* > 0.05). Compared with the blank and NC groups, the miR-182-5p mimic, U0126 and si-ADCY6 groups had a decreased PCNA protein level and proliferation decreased (*P* < 0.05); the protein level of PCNA in the miR-182-5p inhibitor group was increased and proliferation accelerated (*P* < 0.05). There was no significant difference in the cell proliferation in the miR-182-5p inhibitor + si-ADCY6 group and miR-182-5p inhibitor + U0126 group (*P* > 0.05). Compared with the miR-182-5p inhibitor group, the PCNA protein level and the cell proliferation ability were significantly decreased in the miR-182-5p inhibitor + si-ADCY6 and miR-182-5p inhibitor + U0126 groups (all *P* < 0.05). MiR-182-5p could inhibit the proliferation of osteoblasts by inhibiting the Rap1/MAPK signaling pathway, and ADCY6 can promote the proliferation of osteoblasts.

**Figure 7:** The down-regulation of miR-182-5p promotes osteoblast proliferation (**A**) OD value in response to the treatment of miR-182-5p mimic, miR-182-5p inhibitor, si-ADCY6, miR-182-5p inhibitor + si-ADCY6, U0126 or miR-182-5p inhibitor + U0126 measured by MTT assay; (**B**) the gray value of PCNA protein band in response to the treatment of miR-182-5p mimic, miR-182-5p inhibitor, si-ADCY6, miR-182-5p inhibitor + si-ADCY6, U0126 or miR-182-5p inhibitor + U0126; (**C**) PCNA protein level in response to the treatment of miR-182-5p mimic, miR-182-5p inhibitor, si-ADCY6, miR-182-5p inhibitor + si-ADCY6, U0126 or miR-182-5p inhibitor + U0126; *, *P* < 0.05 *vs*. the blank group and the NC group; #, *P* < 0.05 *vs*. the miR-182-5p inhibitor group. NC, negative control; PCNA, proliferating cell nuclear antigen; miR-182-5p, microRNA-182-5p.

### Down-regulated miR-182-5p enhances osteoblast differentiation

The activities of ALP (Figure 8A) and BGP (Figure 8B), as well as the mRNA and protein levels of ALP, BMP2, BGP and COL I (Figure 8C–K) were determined to investigate the effect of miR-182-5p on osteoblast differentiation. There was no significant difference in the levels of ALP and BGP between the blank and NC groups (*P* > 0.05). Compared with the blank and NC groups, the miR-182-5p mimic, siRNA-ADCY6 and U0126 groups had significantly decreased ALP, BMP2 and BGP levels and down-regulated COL I expression (all *P* < 0.05), whereas the miR-182-5p inhibitor group had elevated ALP, BMP2 and BGP levels and up-regulated COL I expression (all *P* < 0.05). There was no significant change in the levels of ALP, BMP2, BGP and COL I in the miR-182-5p inhibitor + si-ADCY6 and miR-182-5p inhibitor + U0126 groups (*P* > 0.05). MiR-182-5p could inhibit the expression of differentiation factors, and ADCY6 could promote the expression of differentiation factors. Down-regulation of miR-182-5p can activate the Rap1/MAPK signaling pathway by targeting ADCY6, thus promoting the differentiation of osteoblasts.

**Figure 8:** Down-regulated miR-182-5p enhances osteoblast differentiation (**A** and **B**) ALP activity and BGP activity in response to the treatment of miR-182-5p mimic, miR-182-5p inhibitor, si-ADCY6, miR-182-5p inhibitor + si-ADCY6, U0126 or miR-182-5p inhibitor + U0126; (**C**) the gray value of ALP, BGP, COL I and BMP2 protein bands in response to the treatment of miR-182-5p mimic, miR-182-5p inhibitor, si-ADCY6, miR-182-5p inhibitor + si-ADCY6, U0126 or miR-182-5p inhibitor + U0126; (**D** and **E**) mRNA and protein levels of COL I in response to the treatment of miR-182-5p mimic, miR-182-5p inhibitor, si-ADCY6, miR-182-5p inhibitor + si-ADCY6, U0126 or miR-182-5p inhibitor + U0126; (**F** and **G**) mRNA and protein levels of ALP in response to the treatment of miR-182-5p mimic, miR-182-5p inhibitor, si-ADCY6, miR-182-5p inhibitor + si-ADCY6, U0126 or miR-182-5p inhibitor + U0126; (**H** and **I**) mRNA and protein levels of BMP2 in response to the treatment of miR-182-5p mimic, miR-182-5p inhibitor, si-ADCY6, miR-182-5p inhibitor + si-ADCY6, U0126 or miR-182-5p inhibitor + U0126. *, *P* < 0.05 *vs*. the blank group and the NC group; #, *P* < 0.05 *vs*. the miR-182-5p inhibitor group. ALP, alkaline phosphatase; BGP, Bone gla protein; COL I, type I collagen; NC, negative control; miR-182-5p, microRNA-182-5p.

### Down-regulated miR-182-5p inhibits cell cycle progression and cell apoptosis of osteoblasts

Flow cytometry was employed to determine the cell cycle distribution (Figure 9A,B) and cell apoptosis (Figure 9C,D). There was no significant difference in the cell cycle distribution and apoptosis rate in the blank and NC groups (*P* > 0.05). Compared with the blank and NC groups, the miR-182-5p mimic, siRNA-ADCY6 and U0126 groups had more cells in the G1 phase and less cells in S phase, as well as significantly increased cell apoptosis (*P* < 0.05). In the miR-182-5p inhibitor group, there were less cells in the G1 phase and increased cells in the S phase, and the cell apoptosis was significantly lower (*P* < 0.05). MiR-182-5p could promote osteoblast apoptosis, while ADCY6 could inhibit osteoblast apoptosis. The down-regulation of miR-182-5p can reverse the apoptosis induced by a low expression of ADCY6, and the Rap1/MAPK signaling pathway inhibitor U0126 can reverse the down-regulated phenotype of miR-182-5p.

**Figure 9:** Down-regulated miR-182-5p inhibits cell cycle progression and cell apoptosis of osteoblasts (**A**) Cell cycle diagram depicting cell progression; (**B**) quantitative analysis for cell cycle progression in response to the treatment of miR-182-5p mimic, miR-182-5p inhibitor, si-ADCY6, miR-182-5p inhibitor + si-ADCY6, U0126 or miR-182-5p inhibitor + U0126; (**C**) flow cytometry map demonstrating cell apoptosis conditions; (**D**) apoptosis rate analysis for cells in response to the treatment of miR-182-5p mimic, miR-182-5p inhibitor, si-ADCY6, miR-182-5p inhibitor + si-ADCY6, U0126 or miR-182-5p inhibitor + U0126; *, *P* < 0.05 *vs*. the blank group and the NC group; #, *P* < 0.05 *vs*. the miR-182-5p inhibitor group; NC, negative control; miR-182-5p, microRNA-182-5p.

## Discussion

OP, a frequently occurring disease, is a metabolic bone disorder that affects millions of individuals worldwide whose high morbidity leads to a high rate of disability, extreme pain and a reduced quality of life [18,19]. MiRNAs have various functions, and it has been reported that they could play a role in bone formation, such as the differentiation of osteoblasts [20]. The therapeutic potentials of miRNAs, including miR-138, miR-338-3p and miR-188, have been proven in OP [21]. Given that each miRNA has many potential functions, it is beneficial for disease treatment to research the mechanism of miRNAs. In the present study, we explored the mechanism of miR-182-5p, ADCY6 and the Rap1/MAPK signaling pathway. Consequently, the present study demonstrates that miR-182-5p regulates the apoptosis and proliferation of osteoblasts through the Rap1/MAPK signaling pathway by negatively targeting the ADCY6 gene.

Initially, we found that in OP, the trabecular bone was thinner, cortical thinning occurred, and the morphological structure was poor with a break. The bone density and area were reduced, the osteoblasts decreased and the osteoclasts increased. Consistent with our study, a study observed through HE staining that there were osteoporotic changes in OP rats, including an increase in the intertrabecular space, thinning of the bone trabeculae and microfractures of the bone trabeculae [22]. Moreover, we found ALN had increased serum calcium, decreased serum phosphorus, an increased BMD and a lower AI of the femur tissues in rats with OP, which indicates that ALN has a therapeutic effect on OP. ALP and COL I expression followed by the maturation of the extracellular matrix in the early stage and ALP, COL and BGP are the main regulatory genes in bone formulation [23]. In many therapies, ALN is currently the most commonly used treatment for OP in patients, with an increasing use of the 70 mg weekly dosages, and the latest formulations of this drug are expected to reduce side effects and increase adherence to the treatment of anti-fractures, aiming at better clinic effects [24]. ALN at a low concentration is beneficial to the formation of bone through promoting the mineralization ability of osteoblasts to a certain extent [25]. According to one experiment, the cell viability was decreased in high concentrations of ALN, indicating that a high dose was cytotoxic, with damage to its therapeutic effect, ultimately resulting in osteonecrosis [26].

According to our research, miR-182-5p directly targets ADCY6 as verified by the dual luciferase reporter gene assay, and following the transfection of miR-182-5p inhibitor, the expressions of ADCY6, ERK1, ERK2, P38 MAPK and Rap1, and the extent of ERK1/2 and P38 MAPK phosphorylation were up-regulated, indicating that miR-182-5p could reduce the expression of ADCY6, thus inhibiting the activation of the Rap1/MAPK signaling pathway. Consistent with our study, there are six predicted target sites in both ADCY6 and miR-182 transcripts, which demonstrates that ADCY6 is a target gene of miR-182 and miR-182 down-regulates the expression of ADCY6 in circadian variation [27]. Interestingly, recent research suggests that the expression of ADCY6 may be directly modulated by miR-182, which is the way ADCY6 participated in circadian rhythm regulation [28]. The MAPK signaling pathway plays a crucial role in regulating osteogenesis, which is a disorder that affects the bones; for example, in ovariectomy-induced bone loss, MAPK was up-regulated [29]. In addition, hsa-miR-205-5p negatively affects osteoblast differentiation via the P38 MAPK signaling pathway [30]. It has been reported that the constitutive activation of the MAPK/ERK and AKT/PKB signaling pathway, as well as the up-regulation of microRNAs, including miR-96, miR-182 and miR-183, were factors that contributed to the inactivation of FOXO1 [31], which indicates that there may be a correlation between miR-182-5p and the Rap1/MAPK pathway.

Furthermore, inhibition of miR-182-5p could promote the ALP and BGP levels and the COL I expression, as well as cell proliferation and differentiation through the Rap1/MAPK signaling pathway via negative regulation of ADCY6. LGR4, a novel RANKL receptor, has been found to suppress osteoclast differentiation and survival induced by RANKL *in vivo* and *in vitro* [32]. A recent publication noted that miR-182 negatively regulates osteoblast differentiation, in which its down-regulation increased osteoblast differentiation [33]. Research has shown that with the down-regulation of p38MAPK and the ERK1/2 signal pathway, the ALP, COL I and BGP expression levels were inhibited [23]. A positive regulation exists between BMP2 induced osteogenic differentiation and p38 MAPK, and the inhibition of MAPK will reduce the differentiation of osteoblasts [34].

In this research, we demonstrate the regulation mechanism of miR-182-5p on osteoblast proliferation and differentiation. The mechanism of miR-182-5p is mediated by the Rap1/MAPK signaling pathway via targeting the ADCY6 gene. We speculate that the miR-182-5p regulated mechanism may be a promising new direction in the development of therapeutic treatments for OP and aims to provide a new basis for the development of targeted therapy. However, we intend to further explore the effects of miR-182-5p on the differentiation of osteoblasts in animals.

## Abbreviations

ADCY6: adenylyl cyclase isoform 6
ALN: alendronate
BCIP: 5-bromo-4-chloro-indolyl-phosphatase
BSA: bovine serum albumin
DAPI: 4′,6-diamidino-2-phenylindole
DMEM: Dulbecco’s Modified Eagle’s Medium
EDTA: ethylenediaminetetraacetic acid
ERK: extracellular signal-regulated kinase
FBS: fetal bovine serum
FITC: fluorescein isothiocyanate
MAPK: mitogen-activated protein kinase
miRNA: microRNA
MUT: mutated
NC: negative control
OD: optical density
OP: osteoporosis
PI: propidium iodide
PNPP: *P*-nitrophenyl phosphate
WT: wild type
